# *Lactobacillus gasseri* SF1183 Affects Intestinal Epithelial Cell Survival and Growth

This article has been retracted.

**DOI:** 10.1371/journal.pone.0069102

**Published:** 2013-07-23

**Authors:** Blanda Di Luccia, Nicola Manzo, Loredana Baccigalupi, Viola Calabrò, Elvira Crescenzi, Ezio Ricca, Alessandra Pollice

**Affiliations:** 1 Department of Biology, University of Naples Federico II-MSA-Via Cinthia, Naples, Italy; 2 Istituto di Endocrinologia ed Oncologia Sperimentale-CNR-via S. Pansini, Naples, Italy; INRA, UR1282, France

## Abstract

It is now commonly accepted that the intestinal microbiota plays a crucial role in the gut physiology and homeostasis, and that both qualitative and quantitative alterations in the compositions of the gut flora exert profound effects on the host’s intestinal cells. In spite of this, the details of the interaction between commensal bacteria and intestinal cells are still largely unknown and only in few cases the molecular mechanisms have been elucidated. Here we analyze the effects of molecules produced and secreted by *Lactobacillus gasseri* SF1183 on human intestinal HCT116 cells. *L. gasseri* is a well known species of lactic acid bacteria, commonly associated to the human intestine and SF1183 is a human strain previously isolated from an ileal biopsy of an healthy volunteer. SF1183 produces and secretes, in a growth phase-dependent way, molecule(s) able to drastically interfere with HCT116 cell proliferation. Although several attempts to purify and identify the bioactive molecule(s) have been so far unsuccessful, a partial characterization has indicated that it is smaller than 3 kDa, thermostable and of proteinaceous nature. *L. gasseri* molecule(s) stimulate a G1-phase arrest of the cell cycle by up-regulation of p21WAF1 rendering cells protected from intrinsic and extrinsic apoptosis. A *L. gasseri*-mediated reduction of apoptosis and of cell proliferation could be relevant in protecting epithelial barrier integrity and helping in reconstituting tissutal homeostasis.

## Introduction

Several recent studies have shown that commensal bacteria, forming the human gut microbiota, establish complex symbiotic interactions with cells of the GastroIntestinal Tract (GIT) and that these interactions significantly contribute to human health [1], [2], [3], [4]. Metagenomic experiments have indicated that the vast majority of the intestinal bacteria belong to two phyla, the Gram-negative Bacteroidetes and the Gram-positive Firmicutes, including the large class of Clostridia and the lactic acid bacteria [5], [6]. However, the composition of the gut microbiota is known to change transiently as a consequence of a variety of factors such as age, diet, enteral infections, pharmacological treatments and immunosuppression [7], [8], [9]. Changes in the microbiota composition have also been associated to several diseases, such as chronic inflammation of the GIT, diabetes and obesity [7], [10], [11], [12], [13], [14], and the oral administration of members of the microbiota has been considered as a potential clinical tool to relieve intestinal dysfunctions [15], [16], [17], [18], [19], [20]. Interest in the beneficial functions of the human microbiota has resulted in the selection of specific strains with putative health-promoting capacities that are recognized as probiotics and are generally selected from isolates of the *Lactobacillus* or *Bifidobacterium* species. Probiotic bacteria have been shown capable to modulate systemic inflammation, cell proliferation and apoptosis, and such properties proposed as useful for future immunomodulatory and cancer prevention strategies [13], [14], [21], [22]. *In vitro* studies have reported the anti-proliferative and pro-apoptotic effects of *Lactobacillus* and *Bifidobacterium* spp. in various cancer cell lines [23], [24], [25], [26], while *in vivo* studies have shown the inhibitory activity of probiotics on liver, bladder and colon tumours in animal models [27], [28], [29], [30].

The molecular mechanisms of interaction between intestinal cells and bacteria have been studied in detail only in few cases and often quorum-sensing autoinducers, communication molecules released by bacteria at high densities, have been shown to modulate host responses either directly or through regulation of bacterial genes involved in gut colonization and host signaling [31], [32]. An example in this context is the quorum-sensing pentapeptide CSF (Competence and Sporulation Factor) of *Bacillus subtilis* that is taken up by Caco-2 cells via the membrane transporter OCTN2 (organic cation transporter 2) and that contributes to eukaryotic cell homeostasis activating survival pathways (p38 MitogenActivatedProteinKinase (MAPK) and protein kinase B) [33]. In other cases the secreted bacterial effectors have not been identified: still unidentified molecules secreted by *Lactobacillus rhamnosus* GG were shown to prevent cytokine-induced apoptosis on two different intestinal cell model systems (YAMC-young adult mouse colon; HT29-colon carcinoma) [34]; molecules secreted by *L. reuteri* were shown to potentiate tumour necrosis factor (TNFα)-induced apoptosis in myeloid leukemia derived cells. In the latter example *L. reuteri* molecules were found to: i) suppress NF-kB activation by inhibiting IkBa degradation; ii) downregulate nuclear factor-kB (NF-kB)-dependent gene products affecting cell proliferation and survival; iii) promote apoptosis by enhancing mitogen-activated protein kinase (MAPK) activities including c-Jun N-terminal kinase and p38 MAPK [35].

*Lactobacillus gasseri* is a well characterized species of low GC gram-positive bacteria, known to represent one of the major homofermentative *Lactobacillus* of the human intestine [36]. We have isolated the SF1183 strain of *L. gasseri* from an ileal biopsy of a human healthy volunteer and, in particular, from the fraction of bacteria tightly associated to the epithelial cells. SF1183 was shown to have antimicrobial activity against a panel of enteropathogens and to form a matrix (biofilm) in standard laboratory as well as in simulated intestinal conditions [36].

This study investigates the effects of molecules produced and secreted by *L. gasseri* SF1183 on colorectal HCT116 cells, both at the molecular and cellular level. Since HCT116 cells are responsive to TNFα-induced apoptosis [37], [38], we tested their response to the presence of *L. gasseri* SF1183 supernatant. Moreover, we extended our analysis to the effects of another inducer of apoptosis to evaluate the specificity of the observed effect.

## Results and Discussion

### The Conditioned Medium (CM) of *L. gasseri* SF1183 Protects HCT116 cells from TNFα Induced Apoptosis

Among the most common features of chronic intestinal inflammations, such as Crohn and irritable bowel diseases (IBDs), is the increase in the production of inflammatory cytokines, epithelial cell apoptosis and immune cell infiltration, leading to disruption of the intestinal epithelial integrity. TNFα is among the cytokines more largely produced under these conditions. It is known to regulate both anti- and pro-apoptotic signaling pathways and determine the cell fate by controlling the balance between the two pathways [39]. To study the effects of molecules secreted by *L. gasseri* on TNFα-induced apoptosis we used the TNFα sensitive HCT116 human colon cancer cells as a model of intestinal epithelial cells [37]. As a marker of apoptosis we followed the proteolytic cleavage of PARP-1, a regulator of the DNA base excision repair pathway essential for the maintenance of genomic integrity and for survival in response to genotoxic insults [40]. PARP-1 is known to be specifically proteolysed by the Caspase 3 to a 24 kDa DNA-binding domain (DBD) and a 89 kDa catalytic fragment during the execution of the apoptotic program [41]. To set up the experimental conditions, HCT116 cells were incubated with 1 nM TNFα for various times and cell extracts analyzed by western blotting with anti-PARP-1 antibody. As shown in Figure 1A, the amount of proteolyzed PARP-1 increased with the time of exposure to TNFα. Therefore we decided to use 8 hours of treatment with 1 nM TNFα to detect either induction or inhibition of PARP cleavage, for all therein experiments involving a TNF-α activation.

**Figure 1:** HCT116 cell response to *L. gasseri* CM with or without TNFα treatment. Western blot with anti-PARP-1 antibody of whole cell extracts from HCT116 cells incubated in (A) complete cell culture medium supplemented or not with TNFα (1 nM) for 2, 8 or 24 hours; (B) complete cell culture medium supplemented or not with CM (20%v/v) for 16 hours before treatment with 1 nM TNFα for 8 hours; (C) complete cell culture medium supplemented or not with TNFα (1 nM) for 8 hours and MDM (20%v/v) or MDM+lactic acid pH4 (20%v/v). After the treatments cells were collected, lysed and protein concentration determined. Equal amount of cell lysates were fractionated on SDS-PAGE and analyzed by western blotting with antibodies against PARP-1. Actin was used as a loading control.

A filter-sterilized conditioned medium (CM) of a *L. gasseri* SF1183 culture was added (20% v/v) to HCT116 cells and incubated for 16 hours. Then, TNFα was added and, after additional 8 hours of incubation, cells were harvested and whole extracts analyzed by western blotting with anti-PARP-1 antibody. As shown in Figure 1B the bacterial CM alone did not have any effect on PARP-1 cleavage while was able to significantly reduce the TNFa-induced proteolytic activation of PARP-1.

*L. gasseri* is a homofermentative bacterium that, therefore, grows producing lactic acid as the only metabolic end-point of carbohydrate metabolism. As a consequence, its growth medium is acidified during growth to reach a final pH value of 4.0. To verify that the reduction in the extent of PARP-1 cleavage was due to secreted molecules and not to the acidification of the growth medium, the same experiment of Figure 1B was performed adding to HCT116 cells the same amount (20% v/v) of the fresh bacterial growth medium (MDM) either at its normal pH (pH 7.0) or acidified to pH 4.0 with lactic acid. As shown in Fig. 1C, both media did not have any effect on TNFα-induced cleavage of PARP-1 suggesting that the CM of *L. gasseri* SF1183 contains molecules with anti-apoptotic activity.

### The CM of *L. gasseri* SF1183 Contains Bioactive Soluble Molecule(s) Secreted During the Stationary Phase of Growth

As a first step toward the characterization of molecule(s) involved in the observed effect, we decided to size-separate the CM of *L. gasseri* by using a 3 kDa molecular mass cut-off filter. As Figure 2A clearly shows we observed bioactivity largely in the filtrate, indicating a small (less than 3 kDa) molecular mass for the effector(s) molecule(s). Further, different enzymatic treatments of the CM indicated that bioactivity is proteinase-K sensitive, suggesting a proteinaceous nature (Figure 2B). After a heat treatment of 30 minutes at 100°C the CM was still able to reduce the TNFa-induced cleavage of PARP-1 at the same extent of untreated CM (Figure 2C), suggesting that the bioactive molecule(s) is not thermolabile. Often bacteria secrete bioactive molecules during their stationary phase of growth. We thus tested the CM of *L. gasseri* cultures at different stages of growth and observed bioactivity produced only in early and late stationary phase of growth (24 and 48 hours of growth, respectively) (Figure 2D). All experiments therein reported have been performed by using the size-fractionated (<3 kDa) CM of a late stationary culture of *L. gasseri* SF1183.

**Figure 2:** *L. gasseri* secretes thermostable, bioactive molecule(s) of proteinaceous nature during the stationary phase of growth. HCT116 cells were incubated in complete cell culture medium supplemented or not with TNFα (1 nM) for 8 hours and with A) CM fractionated with a cut-off of 3 kDa, or B) CM treated with different enzymes [Trypsin, Proteinase K, DNAse I, RNAse A], or C) CM treated at 100°C for 30 minutes, or D) CM of cultures at the indicated phases of growth. After the treatments, cells were collected, lysed and total cell extracts were analyzed by western blotting with antibodies against PARP-1. Actin was used as a loading control. PARP-1 band intensity was evaluated by ImageQuant analysis on at least two different expositions to assure the linearity of each acquisition. Values expressed as ratio with the corresponding actin values and normalised to the reference point (PARP-1 cleavage in medium). Percentage of increase (+) or decrease (–) with respect to the intensity of the reference point are indicated.

### The CM of *L. gasseri* SF1183 Affects Cell Proliferation of HCT116 Cells

To characterize the cellular response to *L. gasseri* secreted molecules, we analyzed HCT116 cell number and viability after growth in presence of CM. Briefly, cells were incubated for 24 hours with CM of *L. gasseri* (20% vol/vol) and then analyzed both for the number of cells by counting in a Burker chamber and for cell viability by MTS assay. As Figure 3A shows, the CM caused a 30% reduction in the number of cells. The MTS assay (Figure 3B) showed a reduction in cell viability of the same order of magnitude.

**Figure 3:** The CM of *L. gasseri* SF1183 affects HCT116 cell number but not cell viability. Proliferating HCT116 cells were incubated in complete cell culture medium supplemented or not with CM (20%v/v). After 24 hours (A) controls (NT) and CM-treated (CM) cells were collected and counted in a Burker chamber; or (B) incubated with 3-(4,5-dimethylthiazol-2-yl)-5-(3-carboxymethoxyphenyl)-2-(4-sulfophenyl)-2H-tetrazolium as a substrate and the absorbance of converted formazan measured at 490 nm.

To get more insights into the cellular response, we looked at the cell-cycle distribution profile and at the expression of cell cycle-related molecular markers in HCT116 cells exposed to TNFα and/or to the CM of *L. gasseri*.

The cell cycle distribution was analyzed by flow cytometry and showed that treatment with TNFα causes a drastic increase in the subG1 cell population (from 4 to 28%) while the pre-treatment of cells with the CM of *L. gasseri* strongly reduced the TNFα induced effect (Figure 4A), thus supporting our previous data indicating a reduction in the extent of PARP-1 cleavage (see Figure 1B, 2B, 2C). Importantly, we found that the CM alone caused a significant increase (up to 18%) in the G1 population of cells with a compensatory decrease in S/G2 cells, indicating that cells were unable to resume the cell cycle at normal phase transit rate (Figure 4A), consistently with previous MTS and proliferation data. This suggests that, indeed, molecules secreted from *L. gasseri* can drastically interfere with proliferation of HCT116 cells, rendering them less prone to TNFα induced apoptosis.

**Figure 4:** The CM of *L. gasseri* SF1183 affects cell proliferation of HCT116 cells. Proliferating HCT116 cells were incubated in complete cell culture medium supplemented or not with CM (20%v/v) and/or TNFα (1 nM). After the treatments, cells were collected and treated for flow-cytometric analysis (A and Fig. S3 in File S1) or western blot (B) with the indicated antibodies.

Expression of the cell cycle markers p21WAF1 and pERKs was also investigated to explore the effects of the CM of *L. gasseri* at the molecular level. p21WAF1 (also known as cyclin-dependent kinase inhibitor 1) is a regulator of cell cycle progression at the S phase that acts as an inhibitor of cyclin-dependent kinase, and occupies a central position in the regulation of the cell cycle in many tissues [42], [43]. Levels of p21WAF1 protein are regulated during the cell cycle at the levels of transcription and protein degradation, although many questions remain on the mechanism of p21 proteolysis [44], [45]. Extracellular signal-regulated kinases (ERK1,2) are members of the MAPK super family that can mediate cell proliferation and apoptosis. Activated (phosphorylated) ERKs, are usually associated with active cell proliferation [46], while p21 increase correlates with a G1 cell cycle arrest [47]. Immunoblots with the appropriate antibodies showed that treatment with CM significantly induced p21WAF independently from TNFα (Figure 4B; compare lanes 1–2 with 3–4) while pERKs expression was inhibited in CM treated cells, strongly supporting the antiproliferative effect of molecule(s) present in *L. gasseri* supernatant.

Altogether these experiments clearly indicate that *L. gasseri* supernatant exerts a cytostatic but not a cytotoxic effect on epithelial colon cells.

### The CM of *L. gasseri* SF1183 Protects HCT116 Cells from Cisplatin Induced Apoptosis

To test whether bioactive molecules present in *L. gasseri* supernatant could exert anti-apoptotic effects against other apoptosis-inducers we preincubated HCT116 cells with CM and then treated them with 30 µM cisplatin to induce the intrinsic apoptotic pathway. As shown in Figure 5A cytofluorimetric analysis indicate that a G1 cell cycle arrest is induced by CM addition which causes cells to be more resistant to cisplatin induced apoptosis. These observations are supported, at the molecular level, with an increase in p21WAF1 levels and a decrease of ERKs activation when CM was added to the cells (Figure 5B, lanes 1,2). Consistently, pretreatment of cells with CM determined a reduction in the extent of PARP-1 cleavage when cells were subjected to cisplatin action (Figure 5B, lanes 3,4).

**Figure 5:** The anti-apoptotic effect of *L. gasseri* is not specific for TNFα-induced apoptosis. Proliferating HCT116 cells were incubated in complete cell culture medium supplemented or not with CM (20%v/v) and/or cisplatin (30 µM). After the treatments, cells were collected and treated for flow-cytometric analysis (A and Fig. S4 in File S1) or western blot (B) with the indicated antibodies.

Altogether our results clearly indicate that probiotic *L. gasseri* protects intestinal epithelial cells from apoptosis induced by inflammatory cytokines or cytotoxic drugs, causing cell cycle arrest.

### Conclusions

The main result of this report is that the conditioned medium of a stationary culture of the human isolate SF1183 of *L. gasseri* contains molecule(s) able to affect cell proliferation of HCT116 cells, protecting them from intrinsic as well as extrinsic, TNFα-induced, apoptosis. Chronic inflammations cause an increase in inflammatory cytokines (such as TNFα), epithelial cell apoptosis and immune cell infiltration, leading to disruption of the intestinal epithelial integrity. Therefore, a reduction of cell proliferation could protect epithelial barrier integrity and help in reconstituting tissutal homeostasis.

The *L. gasseri* molecule(s) responsible of the observed effects is proteinaceous, has a small (less than 3 kDa) size and its synthesis is growth phase-dependent, occuring only in bacterial cells in stationary phase. Those properties are suggestive of bacterial quorum-sensing autoinducers, communication molecules produced at high cell density and known to act as modulator of bacterial host responses [31], [32], [33]. Unfortunately, the definition of the chemical nature of the molecule(s) secreted by *L. gasseri* SF1183 and able to affect HCT116 cells has been so far unsuccessful. The size-fractionated (less than 3 kDa) CM of *L. gasseri* was analyzed by gel filtration chromatography with a Superdex Peptide 10/300 GL (GE Healthcare Life Sciences) column and two main peaks were obtained (Fig. S1 in File S1). Chromatographic fractions containing either one of the two peaks were tested for the ability to reduce the TNFα-induced cleavage of PARP-1 (Fig. S2A in File S1). Only one of the fractions (Fraction 1) was shown to reduce the TNFα-induced cleavage of PARP-1 at the same extent of the unfractionated CM (Fig. S2B in File S1). Unfortunately, attempts to analyze Fraction 1 by mass-spectrometry have been so far unsuccessful, probably because of the minimal concentration of molecules in the fraction. To define the chemical nature of the molecule(s) affecting HCT116 cells and identify its cellular and molecular targets will then be a future and challenging task.

## Materials and Methods

### Bacterial Growth and Preparation of Conditioned Medium

*Lactobacillus gasseri* (SF1183) was grown in MRS broth (Difco, Detroit, MI) for 24 hours at 37°C and the culture diluted and used to inoculate MDM (Glucose 10 g/L, Sodium acetate 5 g/L, KH2PO4 3 g/L, K2HPO4 3 g/L, MgSO4 *7H2O 0.2 g/L, L-Alanine 100 mg/L, L-Arginine 100 mg/L, L-Aspartic acid 200 mg/L, L-Cysteine 200 mg/L, L-Glutamic 200 mg/L, L-Histidine 100 mg/L, L-Isoleucine 100 mg/L, L-Leucine 100 mg/L, L-Lysine 100 mg/L, L-Methionine 100 mg/L, L-Phenylalanine 100 mg/L, L-Serine 100 mg/L, L-Tryptophan 100 mg/L, L-Tyrosine 100 mg/L, L-Valine 100 mg/L, Nicotinic acid 1 mg/L, Pantothenic acid 1 mg/L, Pyridoxal 2 mg/L, Riboflavin 1 mg/L, Cyanocobalamin 1 mg/L, Adenine 10 mg/L, Guanine 10 mg/L, Uracil 10 mg/L) minimal medium. Cells of SF1183 were then grown anaerobically for 48 hours at 37°C. The culture was centrifuged (1000 g for 10 min at RT) and the supernatant (conditioned medium, CM) was filtered-sterilized through a 0.22 µm low-protein binding filter (Millipore, Bedford, MA, US). CM treated with proteases and nucleases was prepared as described above and size fractionated (3-kDa cutoff spin column; Centricon, Millipore). Before treatment with trypsin (GIBCO) or proteinase K (Invitrogen), or DNasi I, or RNasi A (Invitrogen, Life Technology, Monza, Italy) at a final 100 mg/ml concentration for 60 min at 37°C the pH of CM was neutralized with concentrated NaOH (10 N). After the enzymatic treatments CM was acidified to pH 4.0 using concentrated HCl and fractionated as described above to remove the enzymes.

### Cell Culture and Treatment with Bacterial CM

HCT116 cells (ATCC CCL 247) derived from a poorly-differentiated colonic adenocarcinoma and were maintained in RPMI 1640 supplemented with 10% fetal bovine serum and 1% penicillin-streptomycin. Cells were cultured at 37°C in humidified atmosphere of 5% CO_2_. The bacterial CM was employed for the treatment at 20% v/v concentration in complete growth medium. After incubation of 16 hours with CM (20% v/v), TNFα (1 nM) (Millipore, Milan, Italy) or Cisplatin (30 µM) (Sigma Milan, Italy) was added and cells harvested after 8 hours or 24 hours of treatment. Cells were lysed and cell extracts prepared for Western blot and FACS analysis, respectively, as described below.

### SDS-PAGE and Western Immunoblot Analysis

Cells were harvested in lysis buffer (50 mM Tris-HCl pH 7.5, 5 mM EDTA, 150 mM NaCl, 1% NP-40, 1 mM phenylmethylsulfonyl fluoride, 0.5% sodium deoxycholate, and protease inhibitors) and total protein extract prepared as previously described [48]. Briefly, cell lysates were incubated on ice for 40 minutes, and the extracts were centrifuged at 15000 g for 15 minutes to remove cell debris. Protein concentration was determined by the Bio-Rad protein assay (Bio-Rad). After the addition of 2x Laemmli buffer (SIGMA), samples were boiled at 100°C for 5 minutes and resolved by SDS-polyacrylamide gel electrophoresis (10% or 12%). Proteins were transferred to polyvinylidenedifluoride (PVDF) membranes (Millipore Milan, Italy) as previously described [49]. The membranes were blocked in 5% w/v milk buffer (5% w/v non-fat dried milk, 50 mM Tris, 200 mM NaCl, 0,2% Tween 20) and incubated with primary antibody diluted in 5% w/v milk or bovine serum albumine buffer for 2 hours at room temperature or overnight at 4°C. Primary antibodies were anti-rabbit PARP-1 (Cell Signaling, EuroClone, Milan, Italy), anti-rabbit pErks 42/44 (Cell Signaling, EuroClone, Milan, Italy), anti-rabbit p21WAF1 (Santa-Cruz Biotechnology, DBA Milan-Italy), anti-goat β-actin (Santa-Cruz Biotechnology DBA Milan, Italy). Data were visualized by enhanced chemiluminescence method (ECL, GE-Healthcare Milan, Italy) using HRP-conjugated secondary antibody (Santa-Cruz Biotechnology DBA Milan, Italy) incubated 1 hour at room temperature, and analysed by Quantity One ®software of ChemiDoc ^TM^XRS system (Bio-Rad Milan, Italy).

### Cell Growth and Flow Cytometry Analysis

HCT116 cells were plated in 35 mm dishes at the cell density of 2,5×10^5^ cells/plate. For cell growth analysis, cells were cultured in complete growth medium supplemented or not with bacterial CM at 20% v/v concentration for 24 hours. After the treatment, cells were collected and counted in a Burker chamber. Flow cytometry analysis was performed as previously described [50]. Briefly, cells were washed twice with PBS and harvested at 1500 g with 0.05% trypsin in 0.15% Na_2_EDTA. Cells were then centrifuged, washed in PBS, fixed with ice-cold 70% ethanol, and stored overnight at 4°C. Fixed cells were washed in PBS and then incubated with propidium iodide (50 µg/ml) and RNAse A (10 µg/ml) for 30 min at room temperature. Data acquisition was performed using a CyAn ADP Flow Cytometer (Beckman Coulter, Inc., Milano, Italy) and Summit Software.

### MTS Assay

HCT116 cells were cultured at a density of 2,5×10^5^ cells per well in flat bottomed 6-well plates and supplemented or not with CM (20% v/v) for 24 hours. After treatment, CellTiter 96® AQ_UEOUS_ One Solution Reagent (Promega, Madison, WI, US) was added to each well according to the manufacturer’s instructions. After 30 minutes cell viability was determined by measuring the absorbance at 490 nm using a Multiscan spectrum (Thermo Electron Corporation).

## Supporting Information

File S1 Supplemental figures. Figure S1, the CM of L. gasseri was size fractionated with a 3 kDa molecular mass cut-off filter and loaded on a gel filtration chromatographic column (Superdex Peptide 10/300 GL, GE Healthecare Life Sciences). The elution buffer was AMAC 0.3 M. Two main peaks were observed at 220 nm. Figure S2, chromatographic fractions from the experiment of Fig. S1 were tested by western blotting with anti-PARP-1 antibody (A). As a control, cells were also treated with the elution buffer (AMAC 0,3 M). (B) Densitometric analysis of the western blot. PARP-1 band intensity was evaluated by ImageQuant analysis on at least two different expositions to assure the linearity of each acquisition. Values are expressed as ratio with the corresponding actin values and normalised to the reference point (PARP-1 cleavage in medium). Percentage of increase (+) or decrease (–) with respect to the intensity of the reference point are indicated. Figure S3, enlargment of part of Fig. 4 showing the output of the FACS analysis. Figure S4, enlargment of part of Fig. 5 showing the output of the FACS analysis.
(PDF)
